# Effects of Resveratrol Against Induced Metabolic Syndrome in Rats: Role of Oxidative Stress, Inflammation, and Insulin Resistance

**DOI:** 10.1155/2022/3362005

**Published:** 2022-08-11

**Authors:** Doha Reda, Gehad E. Elshopakey, Hebatallah A. Mahgoub, Engy F. Risha, Anmar A. Khan, Bodour S. Rajab, Mohamed E. El-Boshy, Fatma M. Abdelhamid

**Affiliations:** ^1^Department of Clinical Pathology, Faculty of Veterinary Medicine, Mansoura University, Mansoura 35516, Egypt; ^2^Department of Pathology, Faculty of Veterinary Medicine, Mansoura University, Mansoura 35516, Egypt; ^3^Laboratory Medicine Department, Faculty of Applied Medical Sciences, Umm Al-Qura University, Al Abdeyah, P.O. Box 7607, Makkah, Saudi Arabia

## Abstract

Metabolic syndrome (MS) is a serious health problem associated with an increase in risk factors for hepatic steatosis, which is the most common liver disease today. The goal of this study was to investigate the protective effects of resveratrol against metabolic alterations associated with a high-fat high-fructose diet (HFFD). Thirty-two male rats were randomly divided into four equal groups: control (cont.), metabolic syndrome (MS), resveratrol (Res), and metabolic syndrome treated with resveratrol (MS + Res). Resveratrol was administrated orally at a dose of 30 mg/kg·bw, daily. After 10 weeks, body weight, serum biochemical parameters, hepatic oxidative stress, inflammatory markers, as well as mRNA levels of hepatic genes related to lipid metabolism and insulin signaling were measured. In addition, the liver was examined histopathologically to detect lipid deposition. Increased body weight, hepatic dysfunction, dyslipidemia, hepatic insulin resistance, hepatic oxidative and inflammatory stress conditions, upregulation of mRNA expression level of sterol regulatory element binding protein 1-c (SREBP1-c), and downregulation of mRNA expression levels of peroxisome proliferated activated receptor alpha (PPAR*α*) and insulin receptor substrate-2 (IR-S2) were all observed in the MS rats. Hepatic steatosis was confirmed by hematoxylin and eosin and Oil Red O staining. Administration of resveratrol reduced liver steatosis, oxidative stress, and inflammatory state. Also, it improved lipid profile as well as insulin sensitivity and reverted alterations in hepatic mRNA expression levels of the tested genes. Based on these findings, resveratrol could be proposed as a therapeutic approach for MS prevention.

## 1. Introduction

Metabolic syndrome (MS) has been known in the medical literature for more than 80 years. The International Diabetes Foundation (IDF) defines it as a condition characterized by central adiposity and at least two of the following: high triglycerides, low high-density lipoprotein cholesterol, elevated systolic or diastolic blood pressure, and/or diabetes or elevated fasting blood glucose [1]. Metabolic syndrome is closely associated with physical inactivity and increased consumption of foods containing simple sugar carbohydrates and saturated fat [2]. Recent studies have linked excessive consumption of sugar-sweetened beverages, particularly fructose, to increased lipid synthesis and its deposition in the liver tissue [3]. Once the liver gets fatty, it does not respond to the actions of insulin hormone, which include inhibiting production of both glucose and very low density lipoprotein leading to compensatory hyperinsulinemia, mild hyperglycemia, and dyslipidemia [4]. MS is associated with oxidative/antioxidant imbalance, as well as subclinical inflammation, so assessing the oxidative status in MS is helpful in identifying individuals at high risk for metabolic complications [5]. In addition, MS is associated with atherogenic hyperlipemia and dysregulated lipid metabolism [6]. From the foregoing statements, it is crucial to regulate MS through lifestyle management, focusing on improving diet quality, and physical activity, with weight loss as the most important factor to improve all MS characteristics [7].

Several previous literature have pointed out the importance of natural antioxidants, such as plant polyphenols, which in addition to their known anti-inflammatory and antiatherogenic properties have a variety of activities [8–10], such as reducing oxidative stress in cells and increasing metabolic rate, suggesting that they could be used as an antiobesity agent [11]. Resveratrol is a natural polyphenolic substance extracted from the roots of *Polygonum cuspidatum* [12]. It is present in considerable amounts in peanuts, cherries, pistachios, and grapes, with the grape skin having the highest concentration; therefore, red wine is considered an important source of resveratrol [13]. Resveratrol is known for its anti-inflammatory [14], antidiabetic [15], anticancer [16], and cardioprotective properties [17]. It also has antiobesity effects by reducing lipogenesis, increasing lipolysis, and improving glucose homeostasis [18]. Resveratrol is well established for its role as a natural antioxidant and free radical scavenger based on phenolic hydroxyl groups. Therefore, resveratrol is particularly effective in alleviating and curing diseases caused by oxidative stress [19]. It has been shown to improve lipid and glucose metabolism in metabolic tissues, including the liver, resulting in improved glucose uptake and suppressing ectopic lipid deposition [20].

To the authors' knowledge, no former investigations assessed the alleviating effects of resveratrol against dyslipidemia, oxidative hurt, inflammation, and insulin resistance associated with high-fat high-fructose diet (HFFD)–mediated metabolic syndrome in a single study either *in vitro* or *in vivo*. Hence, the present study was undertaken to assess the mechanistic hepatoprotective roles of resveratrol against changes contributed to HFFD-induced metabolic syndrome in rats via evaluation of oxidative/antioxidant molecules, NF-k*β* signaling, lipid-related genes (SREBP1-c/PPAR*α*), and IRS-2.

## 2. Materials and Methods

### 2.1. Chemicals

Resveratrol (purity ≥ 99%, product no. R5010) and dimethyl sulfoxide (DMSO) were obtained from Sigma Aldrich Co. (St. Louis, MO, USA).

### 2.2. Animals, Diets, and Resveratrol Administration

Thirty-two male albino rats, aged 8 weeks and weighing 220–250 g, were obtained from the Zagazig laboratory animal house and kept in plastic cages under conventional environmental conditions. They were fed standard rodent pellet diet and plan water ad libitum. The experiment was carried out following the procedures reviewed and approved by the Faculty of Veterinary Medicine Animal Research Ethical Committee, Mansoura University, Egypt (2021; M/35).

After allowing the rats to acclimate for fourteen days, they were separated into four equal groups of 8 each: control group (cont.), metabolic syndrome group (MS), resveratrol-treated group (Res), and metabolic syndrome group treated with resveratrol (MS + Res). Rats in the control and Res groups were fed a standard chow diet and tap water, while those in the MS and MS + Res groups were fed a high-fat diet according to El-Sayed et al. [21] along with 25% fructose in the drinking water for 10 weeks. Resveratrol was dissolved in a 25% dimethyl sulfoxide (DMSO) solution immediately before use and administrated at a dose of 30 mg/kg·bw via an orogastric tube daily throughout the experiment, based on Andrade et al. [22].

The body weights of the experimental animals were measured every week throughout the experimental period.

### 2.3. Sample Collection and Preparation

After 10 weeks, the rats were anesthetized, and blood samples were drawn from the retro-orbital plexus in clear tubes. Sera were extracted from the blood samples by centrifugation at 1198 × *g* for 10 minutes. They were then separated into aliquots and refrigerated at −20°C for further examinations. The rats were then decapitated, and the liver of each rat was dissected and divided into four portions. The first portion was used to evaluate the lipid peroxidation/antioxidant status of the liver as well as the pro- and anti-inflammatory mediators. It was rinsed in ice-cold saline (20 mM Tris-HCl, 0.14 M NaCl buffer, pH 7.4), homogenized in ice-cold PBS (pH 7.4), and centrifuged at 4°C for 15 minutes at 3000 rpm. The second portion was preserved in RNA for later determination of the mRNA level of hepatic lipid-related genes and IRS-2. The third portion was fixed with 10% purified formalin and stained with hematoxylin and eosin (H&E) for histopathological inspection. The last portion was frozen and stained with Oil Red O (ORO) stain to identify hepatic fat deposits in the liver section.

### 2.4. Assessment of Serum Biochemical Parameters

Serum liver markers, including alanine aminotransferase (ALT) and aspartate aminotransferase (AST), were determined using kits from Human (Wiesbaden, Germany), while alkaline phosphatase (ALP) was measured using kits from ELITech (Paris, France). Total and direct bilirubin were measured colorimetrically using kits from Diamond (Cairo, Egypt). Additionally, total protein and albumin were measured using kits from Stanbio Laboratory (TX, USA). Lipid profile parameters such as triglycerides (TG), total cholesterol (TC), and high-density lipoprotein-cholesterol (HDL-c) were determined using commercial colorimetric assay kits from Spinreact S.A/S.A. U (Sant Esteve de Bas, Spain). Meanwhile, very low density lipoprotein-cholesterol (VLDL-c) and low-density lipoprotein-cholesterol (LDL-c) values were calculated using the Friedewald formula [23]. Serum glucose was measured using kits from Spinreact (Sant Esteve de Bas, Spain), while serum insulin was determined using ready-to-use Rat ELISA kits from Biospes (Chongqing, China). Homeostasis Model Assessment of insulin resistance (HOMA-IR) was evaluated using the following equation [24] R = glucose concentration mmol/l × insulin *μ*IU/ml/22.5. All except insulin were measured spectrophotometrically (spectrophotometer, BM, Germany, 5010), based on standards and protocols provided by manufacturers.

### 2.5. Assessment of Hepatic Lipid Peroxidation/Antioxidant Status

Hepatic lipid peroxide level (malondialdehyde; MDA) and antioxidant parameters such as superoxide dismutase (SOD), catalase (CAT), and reduced glutathione (GSH), as well as serum total antioxidant capacity (sTAC), were all determined using commercially available Bio-Diagnostic ready-made kits (Cairo, Egypt) following the manufacturer's protocol.

### 2.6. Assessment of Hepatic Pro-/Anti-Inflammatory Mediators

Hepatic nuclear factor kappa B (NF-*κ*B) was measured using ready-made Rat ELISA kits from Cusabio (Wuhan, China), while interleukin-10 (IL-10) was determined using Rat ELISA kits from R&D System (Minneapolis, MN, USA), according to the protocols of the tested kits. Bradford's technique was used to adjust the results to total protein levels in the liver samples [25].

### 2.7. Hepatic Gene Expression Analysis

Total liver RNA was extracted using RNeasy Mini Kit from Qiagen (Hilden, Germany), quantified using NanoDrop® ND-1000 spectrophotometer, and used for cDNA synthesis using Revert Aid-Reverse Transcriptase kits from Thermo Fisher Scientific (MA, USA), based on the manufacturer's recommendations. Real-time quantitative PCR assay was performed in Stratagene (MX3005P, USA) using QuantiTect SYBR Green PCR Master Mix (Qiagen). Primer sequences of SREBP1-c [26], PPAR*α* [27], and IRS-2 [28] are listed in Table 1. Stratagene MX3005P software was used to determine amplification curves and cycle threshold (CT) values. Relative mRNA expression levels were calculated using the comparative Ct method (2^−ΔΔCt^) [29] after normalization with those of *β*-actin [30] as a housekeeping gene.

### 2.8. Histopathological Examination of the Liver

Formalin-fixed and alcoholic dehydrated liver sections were embedded in paraffin, cut into 5 *μ*m sections, and stained with H&E. The sectioned tissues were examined for morphological analysis and histological scoring of steatosis, hepatocellular ballooning, and lobular inflammation by light microscopy [31]. To assess lipid accumulation, frozen liver specimens were cut into 10 *μ*m sections using a cryostat (LEICA CM1800) and then fixed and stained with ORO stain [32]. Images were taken randomly from each tissue section using XSZ-07 series of a biological microscope (China) and Apex Minigrab (UK). The ORO-stained sections were automatically analyzed using Image J (https://imagej.nih.gov/ij).

### 2.9. Statistical Analyses

All quantitative values were presented as mean ± standard error of the mean (SEM), tested for normality by Levene test, and statistically assessed by SPSS, version 26 (Chicago, IL, USA). Statistical comparison between the studied groups was performed via one-way ANOVA accompanied by Duncan test and statistical significance was fixed at *P* value lower than 0.05. For histopathological analysis, positive staining areas were statistically analyzed using ANOVA followed by Tukey's multiple comparisons test using *P*value ≤ 0.05, GraphPad Prism for macOS, version 9.2.0 (283).

## 3. Results

### 3.1. Influence of MS and Resveratrol on Body Weight

As depicted in Figure 1, all studied groups had similar mean body weight values at the beginning of the study. Throughout the investigation, the body weight of the MS rats was considerably higher (*P* < 0.05) than that of the control group. Resveratrol treatment in the MS + Res group failed to normalize (*P* > 0.05) the increased body weight with respect to the control group.

### 3.2. Influence of MS and Resveratrol on the Serum Biochemical Parameters

Induction of MS with HFFD resulted in a significant increase (*P* < 0.05) in the serum values of ALT, AST, ALP, total bilirubin, and direct bilirubin, with a marked decrease in the serum levels of total protein and globulin, in comparison with the control group. Resveratrol treatment significantly restored activities of ALT and ALP to normalcy in the MS + Res group compared to the MS group and markedly declined (*P* < 0.05) AST activity, which, however, remained higher than in the control. Meanwhile, it did not significantly (*P* > 0.05) affect the alterations in the total and direct bilirubin, total protein, and globulin serum levels in the MS + Res group compared to those in the MS group (Table 2).

HFFD resulted in hyperlipidemia in the MS group, reflected by a remarkable elevation (*P* < 0.05) in the serum TG, TC, VLDL-c, and LDL-c levels and a significant decline in serum HDL-c (*P* < 0.05) compared to the control rats. Resveratrol treatment significantly declined the TG and VLDL-c concentrations, normalized TC and LDL-c levels, and pronouncedly increased (*P* < 0.05) the HDL-c level in the MS + Res group with respect to the MS group (Table 3).

Table 3 revealed that serum levels of glucose, insulin, and HOMA-IR were dramatically increased (*P* < 0.05) in the MS group compared to the control, indicating decreased glucose tolerance and/or impaired insulin sensitivity. Compared with the MS group, glucose intolerance and insulin resistance were reversed (*P* < 0.05) by resveratrol administration, as noted in the MS + Res group.

### 3.3. Influence of MS and Resveratrol on the Hepatic Lipid Peroxidation/Antioxidant Status

As demonstrated in Figure 2, MS rats exhibited a significant elevation in the hepatic MDA level, while sTAC and hepatic antioxidant parameters (SOD, GSH, and CAT) were substantially depleted compared to the control group. Daily resveratrol administration in the MS + Res group significantly improved (*P* < 0.05) hepatic SOD and GSH values and suppressed hepatic MDA. Furthermore, hepatic CAT activity was numerically increased (*P* < 0.05) in the MS + Res group, meanwhile sTAC was insignificantly (*P* > 0.05) affected compared to the MS group.

### 3.4. Influence of MS and Resveratrol on Hepatic NF-*κ*B and IL-10

As exhibited in Figure 3, the MS rats had a higher level (*P* < 0.05) of hepatic NF-*κ*B and a lower level of IL-10 compared to the control group. Resveratrol administration sustainably diminished (*P* < 0.05) hepatic NF-*κ*B and improved (*P* < 0.05) hepatic IL-10 level in the MS + Res group compared to the MS group, supporting the anti-inflammatory role of resveratrol.

### 3.5. Influence of MS and Resveratrol on Hepatic Lipid-Related Genes and IRS-2

To evaluate the effects of MS and resveratrol on lipid metabolism and insulin signal transduction in the liver, hepatic SREBP1-c, PPAR*α*, and IRS-2 were measured (Figure 4). Significant upregulation of hepatic mRNA expression of SREBP1-c with concomitant downregulation (*P* < 0.05) of hepatic mRNA expression of PPAR*α* and IRS-2 was observed in the MS group compared to the control. The hypolipemic effect of resveratrol was recorded in the MS + Res group, as it suppressed the upregulation (*P* < 0.05) of hepatic mRNA expression of SREBP1-c and a significant upregulation (*P* < 0.05) of hepatic mRNA expression of PPAR*α* relative to the MS group. Additionally, hepatic mRNA expression of IRS-2 was markedly upregulated (*P* < 0.05) with resveratrol administration in the MS + Res group (Figure 4).

### 3.6. Histopathological Examination of Liver Sections Using H&E Staining

Table 4 elucidates the histopathological findings and lesion scoring in the experimental groups. Microvesicular steatosis was evident in the MS and MS + Res groups and affected many acini (predominantly panacinar) (Figures5(a) and 5(b)). It was significantly reduced in the MS + Res group when compared to the MS one. Also, lobular and portal inflammation were reduced (*P* < 0.05) in the MS + Res group versus the MS group (Figures 5(c) and 5(d)). Furthermore, hepatocyte ballooning injury, Mallory's hyaline bodies, megamitochondria, and microgranulomas were evident in the MS and MS + Res groups (Figures 5(e)–5(g)). However, acidophil bodies, pigmented macrophages, glycogenated nuclei, and fibrosis were not observed in either the MS or the MS + Res groups.

### 3.7. Histopathological Examination of Liver Sections Using ORO Staining

Liver sections from the control and Res groups showed small number of hepatocytes with lipid droplets (Figures 6(a) and 6(c)). Sections from MS rats showed diffuse lipid accumulation in most of the hepatocytes (Figure 6(b)). Meanwhile, lipid deposition was reduced in the MS + Res group as compared with MS rats (Figure 6(d)).

## 4. Discussion

This study evaluated the improving actions of resveratrol against overweight, dyslipidemia, insulin resistance, oxidative stress, and inflammation as general features of metabolic syndrome. In the present study, we found that HFFD caused obvious obesity, as evidenced by a gradual increase in body weight after the second week of diet consumption. This may be attributed to the high fructose intake in our MS model as it activates the lipogenic molecules, PPAR*γ* and SREBP1, that promote hepatic FFA inflow and de novo lipogenesis, leading to an increase in caloric and weight gain [33]. In addition, Bjursell et al. [34] associated higher body weight gain in mice fed a western diet with the reduction in locomotor activity. Our result was previously recorded [35, 36]. According to our results, resveratrol could not reduce the excessive body weight gain in the MS + Res group, which is in accordance with previous researchers [37, 38]. However, resveratrol at a high dose of 400 mg/kg/day for 15 and 24 weeks, respectively, in male C57BL/6J mice fed HFD could significantly decrease the final body [39, 40]. This inconsistency could be related to the administration of a high dose of resveratrol for a prolonged period, suggesting that prolonged resveratrol treatment could lead to weight loss.

According to our results, the MS group showed significantly greater body weight than the control group as well as elevated liver injury markers, dyslipidemia, hyperglycemia, and IR. The hepatic tissues of the MS group had a significant increase in the oxidative stress marker, MDA, and inflammatory molecules, NF-*κ*B, while hepatic antioxidant markers, SOD, GSH, and CAT, and anti-inflammatory cytokines, IL-10, as well as sTAC concentration were markedly depleted. Also, RT-PCR revealed that hepatic de novo lipogenesis molecule, SREBP1-c, expression was upregulated, while PPAR*α*, and insulin signaling molecule, IRS-2, were downregulated in the MS group.

MS rats had increased serum ALT, AST, ALP, total bilirubin, and direct bilirubin concentrations, proving that HFFD was able to induce hepatic dysfunction and disorders in bilirubin metabolism. Zhang et al. [41] and Park et al. [35] observed the same results in HFFD-fed rats. These disorders could be related to HFFD-mediated excessive delivery of fatty acids to the liver, resulting in the activation of oxidative stress and inflammatory pathways that promotes the escape of hepatic cellular enzymes [42, 43].

Oxidative damage is a crucial factor in the development of MS and its associated complication that was further indicated in our study by a significant elevation in the hepatic MDA level with a significant decline in hepatic SOD, GSH, CAT, as well as sTAC concentrations, in the MS group. These findings are consistent with earlier researchers [43, 44]. The oxidative stress that occurred in MS might be contributed to increased caloric intake, which leads to increased metabolic load of mitochondria and decreased membrane fluidity, resulting in an overactive electron transport chain that can produce excessive ROS by-products [45, 46]. In addition, MS-associated hyperglycemia provokes more glucose to enter the polyol pathway, causing depletion in NADPH and subsequently decreased hepatic GSH levels [47]. Moreover, HFFD feeding caused hepatic inflammation in the MS group evidenced by increased hepatic inflammatory molecule, NF-*κ*B, level, which may be related to the hepatic lipid buildup that, when subjected to mitochondrial oxidation, produces peroxidation products (ROS) leading to promotion of the NF-*κ*B pathway and subsequently enhancing the production of proinflammatory cytokines [48]. Meanwhile, the decreased anti-inflammatory IL-10 level observed in our study may be linked to T helper 2 malfunction in MS patients [49]. The present biochemical results were further approved histologically in the MS group by the presence of hepatic microvesicular steatosis as well as hepatic portal and lobular inflammation in H&E-stained sections and the presence of lipid droplets of various sizes in ORO-stained sections.

Furthermore, the MS group had significant dyslipidemia evidenced by a significant elevation in the lipid profile parameters [50, 51] that may be attributed to high fructose intake as it can be further metabolized to produce glycerol, or acetyl-CoA that contributes in TG formation and hepatic lipid accumulation [52, 53]. These results were further confirmed by significant upregulation of the hepatic expression of SREBP1-c, which is the most essential transcription factor in de novo lipogenesis, and downregulation of PPAR*α*, a ligand-activated transcriptional factor that controls the expression of genes related to beta-oxidation of fatty acids that corresponded to prior reports [54, 55]. This could be explained by the property of fructose in stimulating SREBP1 expression and suppressing PPAR*α* expression in the rat liver [56]. Likewise, Ide et al. [57] confirmed that excess carbohydrate intake increases hepatic SREBP1-c expression.

MS-induced elevations in the serum glucose, insulin levels, and HOMA-IR imply the development of insulin resistance [58, 59]. This may be related to lipid by-products–mediated activation of the c-Jun-N-terminal kinases signaling pathway in insulin target cells that phosphorylates insulin resistance substrate-1 and 2 at Ser/Thr residues, leading to blocking of the insulin signal [60]. In addition, increased glucose entry into the hexosamine biosynthesis pathway results in the formation of glucosamine and other hexosamine derivatives, which are potent inducers of IR and glucose intolerance [61]. Hepatic insulin resistance state and impairment in insulin signaling were additionally confirmed in our MS model by a remarkable reduction in the hepatic expression of IRS-2 [62]. Prior studies confirmed the effect of HFD in lessening hepatic IRS-2 mRNA expression levels in rodent animal models [63–65].

Resveratrol has protective and curative effects on liver function, dyslipidemia, oxidative stress, inflammation, insulin resistance, and histological liver damage. The protective role of Res could be attributed to its ability to improve lipid metabolism and interfere with lipid deposition in the liver by inhibiting SREBP1-c and enhancing PPAR*α* hepatic expression [22, 66]. Besides, it plays a role in shifting lipid metabolism toward oxidation [67]. This fact was further confirmed by Wang et al. [68], who claimed that Res inhibited SREBP1 expression in the cell model of steatosis. In addition, Wu et al. [69] revealed that Res administration at a dose of 400 mg/kg diet for 12 weeks restored HFD-mediated reduction in the hepatic expression of PPAR*α* in male C57BL/6J mice. Also, it has been reported that Res attenuated mRNA expression level of HMG-CoA reductase resulting in decreased hepatic cholesterol biosynthesis [70]. These findings were further confirmed histopathologically by a significant decrease in both steatosis degree and the number of lipid droplets in the MS + RSV group on Res treatment.

In line with Bagul et al. [71], Res administration markedly decreased serum levels of glucose, insulin, and HOMA-IR index in the MS + Res group. This may be contributed to the role of Res in protecting pancreatic *β* cells from free radical damage and deleterious cytokine [72]. Besides its vital role in decreasing adiposity [15], the ability of Res to improve insulin sensitivity was further confirmed in our study by upregulation of the expression of IRS-2 in our MS model, which was previously demonstrated in rats fed high-fructose corn syrup [73].

According to our data, Res has been demonstrated to possess antioxidant potential, which was documented in earlier studies [71, 74]. This may be linked to its ability to significantly decrease MDA hepatic levels and increase SOD and GSH hepatic values. Furthermore, Res showed anti-inflammatory properties as it largely reverted the changes in hepatic NF-*κ*B and IL-10 levels, which corresponded to prior reports [75, 76]. This may be referred to the fact that Res can suppress the translocation of NF-*κ*B to the nucleus and subsequently the production of the proinflammatory cytokines [77].

## 5. Conclusions

HFFD consumption was implicated in the development of MS, which was linked with dyslipidemia, insulin resistance, hepatic oxidative stress, inflammatory condition, and alteration in hepatic expression of genes involved in lipid metabolism and insulin signaling transduction. In addition, we concluded that resveratrol showed partial improvements in obesity, metabolic profiles, PPARs, SREBP1, inflammation, and oxidative stress. However, more studies are needed to measure the metabolic effects and therapeutic values of resveratrol for the treatment of MS.

## Figures and Tables

**Figure 1:** Body weight (g) of the studied groups during the experimental period. Data are expressed as means ± S.E.M. Mean with dissimilar superscript letter differed significantly. Cont., control; MS, metabolic syndrome; Res, resveratrol.

**Figure 2:** Effects of resveratrol on HFFD-induced metabolic changes in the hepatic oxidative stress and antioxidant parameters: (a) MDA (malondialdehyde); (b) SOD (superoxide dismutase); (c) GSH (reduced glutathione); (d) CAT (catalase); and (e) sTAC (serum total antioxidant capacity). Data (*n* = 8) are expressed as means ± S.E.M. Cont., control; MS, metabolic syndrome; Res, resveratrol. The mean superscripts with different letters varied significantly (*P* < 0.05).

**Figure 3:** Effects of resveratrol on HFFD-induced metabolic changes in hepatic (a) NF-*κ*B (nuclear factor kappa) and (b) IL-10 (interleukin-10). Data are expressed as means ± S.E.M. Cont., control; MS, metabolic syndrome; Res, resveratrol. The mean superscripts with different letters varied significantly (*P* < 0.05).

**Figure 4:** Effects of resveratrol on HFFD-induced metabolic changes in hepatic mRNA expression levels of (a) SREBP1-c; (b) PPAR*α*; and (c) IRS-2. Data are expressed as means ± S.E.M. Cont., control; MS, metabolic syndrome; Res, resveratrol. SREBP1-c, sterol regulatory element binding protein 1-c; PPAR*α*, peroxisome proliferated activated receptor alpha; IRS-2, insulin receptor substrate-2. The mean superscripts with different letters varied significantly (*P* < 0.05).

**Figure 5:** Histopathological examinations of liver sections using H&E: (a) hepatic panacinar steatosis (10×); (b) hepatocyte microvesicular steatosis (40×); (c) hepatic lobular inflammation (10×); (d) hepatic portal inflammation (10×); (e) Mallory-Denk bodies (arrows) in ballooned hepatocytes (40×); (f) hepatocyte megamitochondria (40×); and (g) hepatic microgranuloma (Mi) (10×).

**Figure 6:** Histopathological examinations of liver sections using Oil Red O staining: (a) cont. group: showing only a few hepatocytes that have tiny lipid droplets; (b) MS group showing diffusely mixed sizes of lipid droplets in most of the hepatocytes; (c) Res group showing a small number of hepatocytes with lipid droplets; (d) MS + Res group showing decreased number of lipid droplets in the hepatic tissue when they are compared with the MS group; and (e) mean positive area percentage ± SEM in each group. Data were analyzed using one-way ANOVA followed by Tukey's test for group comparison. ns = not significant. ^*∗*^*P* value ≤ 0.05; ^*∗∗*^*P* value ≤ 0.01; ^*∗∗∗*^*P* value ≤ 0.001; ^*∗∗∗∗*^ = *P* value ≤ 0.0001.

**Table 1:** Primer sequences for RT-PCR.

Gene	Primer sequence (5′-3′)
Rat *β*-actin	TCCTCCTGAGCGCAAGTACTCT
	GCTCAGTAACAGTCCGCCTAGAA

SREBP1-c	AGGAGGCCATCTTGTTGCTT
	GTTTTGACCCTTAGGGCAGC

PPAR *α*	TCTGTGGGCTCACTGTTCT
	AGGGCTCATCCTGTCTTTG

IRS-2	GAAGCGGCTAAGTCTCATGG
	GACGGTGGTGGTAGAGGAAA

**Table 2:** Effect of resveratrol on the serum liver function indicators in HFFD-induced MS rats.

Parameters	Experimental groups			
	Cont.	MS	Res	MS + Res
ALT (U/L)	44.80 ± 2.15^b^	59.20 ± 3.02^a^	43.60 ± 2.87^b^	47.20 ± 3.51^b^
AST (U/L)	53.80 ± 2.31^c^	76.80 ± 2.21^a^	55.50 ± 2.20^c^	63.60 ± 2.44^b^
ALP (U/L)	333.14 ± 18.73^b^	424.74 ± 14.77^a^	322.56 ± 13.38^b^	345.10 ± 11.03^b^
Total bilirubin (mg/dl)	0.22 ± 0.19^b^	0.40 ± 0.02^a^	0.20 ± 0.03^b^	0.37 ± 0.02^a^
Direct bilirubin (mg/dl)	0.13 ± 0.03^b^	0.28 ± 0.02^a^	0.13 ± 0.01^b^	0.23 ± 0.01^a^
Indirect bilirubin (mg/dl)	0.09 ± 0.02^ab^	0.12 ± 0.01^ab^	0.07 ± 0.02^b^	0.14 ± 0.02^a^
Total protein (g/dl)	9.41 ± 0.20^a^	7.72 ± 0.06^b^	9.24 ± 0.37^a^	8.00 ± 0.17^b^
Albumin (g/dl)	4.73 ± 0.26^a^	4.39 ± 0.10^a^	4.66 ± 0.10^a^	4.60 ± 0.15^a^
Globulin (g/dl)	4.68 ± 0.12^a^	3.33 ± 0.12^b^	4.58 ± 0.34^a^	3.40 ± 0.09^b^
A/G ratio	1.02 ± 0.76^b^	1.32 ± 0.04^a^	1.04 ± 0.09^b^	1.35 ± 0.06^a^

Values are presented as mean ± SEM for eight rats per group. Means with different superscripts in the same row differed significantly, *P* < 0.05. Cont.: control; MS: metabolic syndrome; Res: resveratrol; MS + Res: metabolic syndrome + resveratrol; ALT: alanine aminotransferase; AST: aspartate aminotransferase; ALP: alkaline phosphatase; A/G ratio: albumin/globulin ratio.

**Table 3:** Effect of resveratrol on the serum lipid profile and hemostatic glucose parameters in HFFD-induced MS rats.

Parameters	Experimental groups			
	Cont.	MS	Res	MS + Res
TG (mg/dl)	182.78 ± 4.88^c^	262.06 ± 9.51^a^	183.70 ± 3.71^c^	236.01 ± 6.97^b^
TC (mg/dl)	182.99 ± 2.46^b^	199.20 ± 3.34^a^	180.80 ± 2.35^b^	185.40 ± 2.50^b^
VLDL-c (mg/dl)	36.55 ± 0.98^c^	52.41 ± 1.23^a^	36.74 ± 0.74^c^	47.20 ± 1.39^b^
LDL-c (mg/dl)	70.44 ± 4.80^b^	86.54 ± 4.79^a^	66.86 ± 2.31^b^	70.20 ± 3.47^b^
HDL-c (mg/dl)	76.00 ± 1.76^a^	60.25 ± 1.24^c^	77.20 ± 2.52^a^	68.00 ± 1.14^b^
Glucose (mg/dl)	94.55 ± 3.71^c^	141.49 ± 5.01^a^	99.45 ± 2.10^c^	126.69 ± 3.16^b^
Insulin (*μ*IU/ml)	5.37 ± 0.12^c^	8.20 ± 0.17^a^	5.33 ± 0.18^c^	6.80 ± 0.53^b^
HOMA-IR	1.21 ± 0.04^c^	2.82 ± 0.05^a^	1.27 ± 0.03^c^	2.18 ± 0.19^b^

Values are presented as mean ± SEM for eight rats per group. Means with different superscripts in the same row differ significantly, *P* < 0.05. Cont.: control; MS: metabolic syndrome; Res: resveratrol; MS + Res: metabolic syndrome + resveratrol. TG: triglyceride; TC: total cholesterol; VLDL-c: very low density lipoprotein-cholesterol; LDL-c: low-density lipoprotein-cholesterol; HDL-c: high-density lipoprotein-cholesterol; HOMA-IR: homeostasis model assessment for insulin resistance.

**Table 4:** Hepatic histopathological alterations and lesion scoring in HFFD-induced MS rats.

Item	Definition	Score/code	MS	MS + Res
Steatosis grade	Low- to medium-power evaluation of parenchymal involvement by steatosis			
	<5%	0		
	5%–33%	1		+
	>33%–66%	2	+	
	>66%	3		

Location	Predominant distribution pattern			
	Zone 3	0		
	Zone 1	1		
	A zonal	2		
	Panacinar	3	+	+

Microvesicular steatosis	Contiguous patches			
	Not present	0		
	Present	1	+	+
Fibrosis stage	None	0	+	+
Inflammation	Overall assessment of all inflammatory foci			

Lobular inflammation	No foci	0		
	<2 foci per 200× field	1		+
	2–4 foci per 200× field	2	+	
	>4 foci per 200× field	3		

Portal inflammation	Assessed from low magnification			
	None to minimal	0		+
	Greater than minimal	1	+	

Microgranulomas	Small aggregates of macrophages			
	Absent	0		
	Present	1	+	+

Liver cell injury ballooning	None	0		
	Few balloon cells	1		
	Many cells/prominent ballooning	2	+	+

Acidophil bodies	None to rare	0	+	+
	Many	1		

Pigmented macrophages	None to rare	0	+	+
	Many	1		

Megamitochondria	None to rare	0		
	Many	1	+	+
Other findings				

Mallory's hyaline	Visible on routine stains			
	None to rare	0		
	Many	1	+	+

Glycogenated nuclei	Contiguous patches			
	None to rare	0	+	+
	Many	1		

## Data Availability

The data used to support the findings of this study are included within the article.

## References

[1] Cherniack E. P. (2011). Polyphenols: planting the seeds of treatment for the metabolic syndrome. *Nutrition*.

[2] Alam M. A., Kauter K., Brown L. (2013). Naringin improves diet-induced cardiovascular dysfunction and obesity in high carbohydrate, high fat diet-fed rats. *Nutrients*.

[3] Moore J. B., Gunn P. J., Fielding B. A. (2014). The role of dietary sugars and de novo lipogenesis in non-alcoholic fatty liver disease. *Nutrients*.

[4] Yki-Järvinen H. (2010). Liver fat in the pathogenesis of insulin resistance and type 2 diabetes. *Digestive Diseases*.

[5] Hopps E., Noto D., Caimi G., Averna M. (2010). A novel component of the metabolic syndrome: the oxidative stress. *Nutrition, Metabolism, and Cardiovascular Diseases*.

[6] Fonseca V. A. (2005). The metabolic syndrome, hyperlipidemia, and insulin resistance. *Clinical Cornerstone*.

[7] Batista-Jorge G., Barcala-Jorge A., Silveira M. (2020). Oral resveratrol supplementation improves metabolic syndrome features in obese patients submitted to a lifestyle-changing program. *Life Sciences*.

[8] Elmahallawy E. K., Elshopakey G. E., Saleh A. A. (2020). S-methylcysteine (SMC) ameliorates intestinal, hepatic, and splenic damage induced by cryptosporidium parvum infection via targeting inflammatory modulators and oxidative stress in Swiss albino mice. *Biomedicines*.

[9] Elshopakey G. E., Elazab S. T. J. V. S. (2021). Cinnamon aqueous extract attenuates diclofenac sodium and oxytetracycline mediated hepato-renal toxicity and modulates oxidative stress, cell apoptosis, and inflammation in male albino rats. *Veterinary Sciences*.

[10] Osama A., Engy R., Gehad E. J. A. V. A. S. (2014). Immunomodulatory effect of artichoke (*Cynara scolymus*) on carbon tetrachloride induced immunosuppression in rats. *Annals of Veterinary and Animal Science*.

[11] Rubio-Ruiz M. E., Guarner-Lans V., Cano-Martínez A. (2019). Resveratrol and quercetin administration improves antioxidant defenses and reduces fatty liver in metabolic syndrome rats. *Molecules*.

[12] Huang X.-T., Li X., Xie M.-L. (2019). Resveratrol: review on its discovery, anti-leukemia effects and pharmacokinetics. *Chemico-Biological Interactions*.

[13] Guerrero R. F., Garcia-Parrilla M. C., Puertas B., Cantos-Villar E. (2009). Wine, resveratrol and health: a review. *Natural Product Communications*.

[14] Meng X., Zhou J., Zhao C.-N., Gan R.-Y., Li H.-B. (2020). Health benefits and molecular mechanisms of resveratrol: a narrative review. *Foods*.

[15] Szkudelski T., Szkudelska K. (2011). Anti-diabetic effects of resveratrol. *Annals of the New York Academy of Sciences*.

[16] Signorelli P., Ghidoni R. (2005). Resveratrol as an anticancer nutrient: molecular basis, open questions and promises. *The Journal of Nutritional Biochemistry*.

[17] Hao H. D., He L. R. (2004). Mechanisms of cardiovascular protection by resveratrol. *Journal of Medicinal Food*.

[18] Méndez-del Villar M., González-Ortiz M., Martínez-Abundis E., Pérez-Rubio K. G., Lizárraga-Valdez R. (2014). Effect of resveratrol administration on metabolic syndrome, insulin sensitivity, and insulin secretion. *Metabolic Syndrome and Related Disorders*.

[19] Queiroz A. N., Gomes B. A. Q., Moraes W. M., Borges R. S. (2009). A theoretical antioxidant pharmacophore for resveratrol. *European Journal of Medicinal Chemistry*.

[20] Gong L., Guo S., Zou Z. (2020). Resveratrol ameliorates metabolic disorders and insulin resistance in high-fat diet-fed mice. *Life Sciences*.

[21] El-Sayed M. M., Ghareeb D. A., Talat H. A., Sarhan E. M. (2013). High fat diet induced insulin resistance and elevated retinol binding protein 4 in female rats; treatment and protection with *Berberis vulgaris* extract and vitamin A. *Pakistan Journal of Pharmaceutical Sciences*.

[22] Andrade J. M. O., Paraíso A. F., de Oliveira M. V. M. (2014). Resveratrol attenuates hepatic steatosis in high-fat fed mice by decreasing lipogenesis and inflammation. *Nutrition*.

[23] Friedewald W. T., Levy R. I., Fredrickson D. S. (1972). Estimation of the concentration of low-density lipoprotein cholesterol in plasma, without use of the preparative ultracentrifuge. *Clinical Chemistry*.

[24] Matthews D. R., Hosker J. P., Rudenski A. S., Naylor B. A., Treacher D. F., Turner R. C. (1985). Homeostasis model assessment: insulin resistance and *β*-cell function from fasting plasma glucose and insulin concentrations in man. *Diabetologia*.

[25] Bradford M. M. (1976). A rapid and sensitive method for the quantitation of microgram quantities of protein utilizing the principle of protein-dye binding. *Analytical Biochemistry*.

[26] Ren L., Sun D., Zhou X. (2019). Chronic treatment with the modified Longdan Xiegan Tang attenuates olanzapine-induced fatty liver in rats by regulating hepatic de novo lipogenesis and fatty acid beta-oxidation-associated gene expression mediated by SREBP-1c, PPAR-alpha and AMPK-alpha. *Journal of Ethnopharmacology*.

[27] Ding L., Li J., Song B. (2014). Andrographolide prevents high-fat diet–induced obesity in C57BL/6 mice by suppressing the sterol regulatory element-binding protein pathway. *Journal of Pharmacology and Experimental Therapeutics*.

[28] Kanuri G., Landmann M., Priebs J. (2016). Moderate alcohol consumption diminishes the development of non-alcoholic fatty liver disease (NAFLD) in ob/ob mice. *European Journal of Nutrition*.

[29] Livak K. J., Schmittgen T. D. (2001). Analysis of relative gene expression data using real-time quantitative PCR and the 2−ΔΔCT method. *Methods*.

[30] Banni M., Messaoudi I., Said L., El Heni J., Kerkeni A., Said K. (2010). Metallothionein gene expression in liver of rats exposed to cadmium and supplemented with zinc and selenium. *Archives of Environmental Contamination and Toxicology*.

[31] Kleiner D. E., Brunt E. M., van Natta M. (2005). Design and validation of a histological scoring system for nonalcoholic fatty liver disease. *Hepatology*.

[32] Green H., Kehinde O. (1974). Sublines of mouse 3T3 cells that accumulate lipid. *Cell*.

[33] Refaat B., Abdelghany A. H., Ahmad J. (2022). Vitamin D3 enhances the effects of omega-3 oils against metabolic dysfunction-associated fatty liver disease in rat. *BioFactors*.

[34] Bjursell M., Gerdin A.-K., Lelliott C. J. (2008). Acutely reduced locomotor activity is a major contributor to western diet-induced obesity in mice. *American Journal of Physiology - Endocrinology and Metabolism*.

[35] Park E.-J., Lee Y.-S., Kim S. M. (2020). Beneficial effects of Lactobacillus plantarum strains on non-alcoholic fatty liver disease in high fat/high fructose diet-fed rats. *Nutrients*.

[36] Qin L., Zhao Y., Zhang B., Li Y. (2018). Amentoflavone improves cardiovascular dysfunction and metabolic abnormalities in high fructose and fat diet-fed rats. *Food & Function*.

[37] Jiang M., Li X., Yu X. (2017). Oral administration of resveratrol alleviates osteoarthritis pathology in C57BL/6J mice model induced by a high-fat diet. *Mediators of Inflammation*.

[38] Tian Y., Ma J., Wang W. (2016). Resveratrol supplement inhibited the NF-*κ*B inflammation pathway through activating AMPK*α*-SIRT1 pathway in mice with fatty liver. *Molecular and Cellular Biochemistry*.

[39] Lagouge M., Argmann C., Gerhart-Hines Z. (2006). Resveratrol improves mitochondrial function and protects against metabolic disease by activating SIRT1 and PGC-1*α*. *Cell*.

[40] Zhang J., Chen L., Zheng J. (2012). The protective effect of resveratrol on islet insulin secretion and morphology in mice on a high-fat diet. *Diabetes Research and Clinical Practice*.

[41] Zhang J., Zhao L., Cheng Q. (2018). Structurally different flavonoid subclasses attenuate high-fat and high-fructose diet induced metabolic syndrome in rats. *Journal of Agricultural and Food Chemistry*.

[42] Hussein S. A., Abdel-Magid A. D., Fareed F. A. E. (2017). Biochemical effect of resveratrol on lipids profile and hepatic oxidative stress in experimentally induced obesity in female rats. *Benha Veterinary Medical Journal*.

[43] Khlifi R., Dhaouefi Z., Toumia I. B. (2020). Erica multiflora extract rich in quercetin-3-O-glucoside and kaempferol-3-O-glucoside alleviates high fat and fructose diet-induced fatty liver disease by modulating metabolic and inflammatory pathways in Wistar rats. *The Journal of Nutritional Biochemistry*.

[44] Cui B., Liu S., Lin X. (2011). Effects of lycium barbarum aqueous and ethanol extracts on high-fat-diet induced oxidative stress in rat liver tissue. *Molecules*.

[45] Novelli E. L. B., Diniz Y. S., Galhardi C. M. (2007). Anthropometrical parameters and markers of obesity in rats. *Laboratory Animals*.

[46] Rani V., Deep G., Singh R. K., Palle K., Yadav U. C. S. (2016). Oxidative stress and metabolic disorders: pathogenesis and therapeutic strategies. *Life Sciences*.

[47] Chung S. S. M., Ho E. C. M., Lam K. S. L., Chung S. K. (2003). Contribution of polyol pathway to diabetes-induced oxidative stress. *Journal of the American Society of Nephrology*.

[48] Boden G., She P., Mozzoli M. (2005). Free fatty acids produce insulin resistance and activate the proinflammatory nuclear factor-*κ*b pathway in rat liver. *Diabetes*.

[49] Cano Barquilla P., Pagano E. S., Jiménez-Ortega V., Fernández-Mateos P., Esquifino A. I., Cardinali D. P. (2014). Melatonin normalizes clinical and biochemical parameters of mild inflammation in diet-induced metabolic syndrome in rats. *Journal of Pineal Research*.

[50] Aguilera-Mendez A., Hernández-Equihua M. G., Rueda-Rocha A. C. (2018). Protective effect of supplementation with biotin against high-fructose-induced metabolic syndrome in rats. *Nutrition Research*.

[51] Panchal S. K., Poudyal H., Brown L. (2012). Quercetin ameliorates cardiovascular, hepatic, and metabolic changes in diet-induced metabolic syndrome in rats. *Journal of Nutrition*.

[52] Abdullah M. M., Riediger N. N., Chen Q. (2009). Effects of long-term consumption of a high-fructose diet on conventional cardiovascular risk factors in Sprague-Dawley rats. *Molecular and Cellular Biochemistry*.

[53] Rutledge A. C., Adeli K. (2008). Fructose and the metabolic syndrome: pathophysiology and molecular mechanisms. *Nutrition Reviews*.

[54] Inamdar S., Joshi A., Malik S., Boppana R., Ghaskadbi S. (2019). Vitexin alleviates non-alcoholic fatty liver disease by activating AMPK in high fat diet fed mice. *Biochemical and Biophysical Research Communications*.

[55] Yin Y., Yu Z., Xia M., Luo X., Lu X., Ling W. (2012). Vitamin D attenuates high fat diet–induced hepatic steatosis in rats by modulating lipid metabolism. *European Journal of Clinical Investigation*.

[56] Nagai Y., Nishio Y., Nakamura T., Maegawa H., Kikkawa R., Kashiwagi A. (2002). Amelioration of high fructose-induced metabolic derangements by activation of PPAR*α*. *American Journal of Physiology - Endocrinology and Metabolism*.

[57] Ide T., Shimano H., Yahagi N. (2004). SREBPs suppress IRS-2-mediated insulin signalling in the liver. *Nature Cell Biology*.

[58] Ehrampoush E., Homayounfar R., Davoodi S. H., Zand H., Askari A., Kouhpayeh S. A. (2016). Ability of dairy fat in inducing metabolic syndrome in rats. *SpringerPlus*.

[59] Gancheva S., Zhelyazkova-Savova M., Galunska B., Chervenkov T. (2015). Experimental models of metabolic syndrome in rats. *Scripta Scientifica Medica*.

[60] Feng J., Lu S., Ou B. (2020). The role of JNk signaling pathway in obesity-driven insulin resistance-driven insulin resistance. *Diabetes, Metabolic Syndrome and Obesity: Targets and Therapy*.

[61] Schaalan M., El-Abhar H. S., Barakat M., El-Denshary E. S. (2009). Westernized-like-diet-fed rats: effect on glucose homeostasis, lipid profile, and adipocyte hormones and their modulation by rosiglitazone and glimepiride. *Journal of Diabetes and Its Complications*.

[62] Aragno M., Tomasinelli C. E., Vercellinatto I. (2009). SREBP-1c in nonalcoholic fatty liver disease induced by western-type high-fat diet plus fructose in rats. *Free Radical Biology and Medicine*.

[63] Qiu X., Gao D.-H., Xiang X. (2015). Ameliorative effects of lutein on non-alcoholic fatty liver disease in rats. *World Journal of Gastroenterology*.

[64] Xing L.-J., Zhang L., Liu T., Hua Y.-Q., Zheng P.-Y., Ji G. (2011). Berberine reducing insulin resistance by up-regulating IRS-2 mRNA expression in nonalcoholic fatty liver disease (NAFLD) rat liver. *European Journal of Pharmacology*.

[65] Yang P., Liang Y., Luo Y. (2019). Liraglutide ameliorates nonalcoholic fatty liver disease in diabetic mice via the IRS2/PI3K/Akt signaling pathway. *Diabetes, Metabolic Syndrome and Obesity: Targets and Therapy*.

[66] Huang Y., Lang H., Chen K. (2020). Resveratrol protects against nonalcoholic fatty liver disease by improving lipid metabolism and redox homeostasis via the PPAR*α* pathway. *Applied Physiology Nutrition and Metabolism*.

[67] Alberdi G., Rodríguez V. M., Macarulla M. T., Miranda J., Churruca I., Portillo M. P. (2013). Hepatic lipid metabolic pathways modified by resveratrol in rats fed an obesogenic diet. *Nutrition*.

[68] Wang G.-L., Fu Y.-C., Xu W.-C., Feng Y.-Q., Fang S.-R., Zhou X.-H. (2009). Resveratrol inhibits the expression of SREBP1 in cell model of steatosis via Sirt1–FOXO1 signaling pathway. *Biochemical and Biophysical Research Communications*.

[69] Wu J., Li Y., Yu J. (2020). Resveratrol attenuates high-fat diet induced hepatic lipid homeostasis disorder and decreases m6A RNA methylation. *Frontiers in Pharmacology*.

[70] Cho I. J., Ahn J. Y., Kim S., Choi M. S., Ha T. Y. (2008). Resveratrol attenuates the expression of HMG-CoA reductase mRNA in hamsters. *Biochemical and Biophysical Research Communications*.

[71] Bagul P. K., Middela H., Matapally S. (2012). Attenuation of insulin resistance, metabolic syndrome and hepatic oxidative stress by resveratrol in fructose-fed rats. *Pharmacological Research*.

[72] Rehman K., Saeed K., Munawar S. M., Akash M. S. H. (2018). Resveratrol regulates hyperglycemia-induced modulations in experimental diabetic animal model. *Biomedicine & Pharmacotherapy*.

[73] Sadi G., Ergin V., Yilmaz G. (2015). High-fructose corn syrup-induced hepatic dysfunction in rats: improving effect of resveratrol. *European Journal of Nutrition*.

[74] Banez M. J., Geluz M. I., Chandra A. (2020). A systemic review on the antioxidant and anti-inflammatory effects of resveratrol, curcumin, and dietary nitric oxide supplementation on human cardiovascular health. *Nutrition Research*.

[75] Chang C.-C., Chang C.-Y., Huang J.-P., Hung L.-M. (2012). Effect of resveratrol on oxidative and inflammatory stress in liver and spleen of streptozotocin-induced type 1 diabetic rats. *The Chinese Journal of Physiology*.

[76] Hajighasem A., Farzanegi P., Mazaheri Z. (2019). Effects of combined therapy with resveratrol, continuous and interval exercises on apoptosis, oxidative stress, and inflammatory biomarkers in the liver of old rats with non-alcoholic fatty liver disease. *Archives of Physiology and Biochemistry*.

[77] Ma C., Wang Y., Dong L., Li M., Cai W. (2015). Anti-inflammatory effect of resveratrol through the suppression of NF-kappa B and JAK/STAT signaling pathways. *Acta Biochimica et Biophysica Sinica*.

